The article "Predicting Risk of Insulin Resistance in a Chinese Population with Polycystic Ovary Syndrome: Designing and Testing a New Predictive Nomogram" was retracted in 2024. Reasons: signs of a paper mill; suspected computer-generated content; unreliable results or conclusions; concerns about the data.

# Predicting Risk of Insulin Resistance in a Chinese Population with Polycystic Ovary Syndrome: Designing and Testing a New Predictive Nomogram

**DOI:** 10.1155/2020/8031497

**Published:** 2020-06-13

**Authors:** Feng Jiang, Ke Wei, Wenjun Lyu, Chuyan Wu

**Affiliations:** ^1^Pediatric Department, The First Affiliated Hospital of Nanjing Medical University, Nanjing 210000, China; ^2^Neonatal Department, Obstetrics and Gynecology Hospital of Fudan University, No. 419 Fangxie Road, Huangpu District, Shanghai 200011, China; ^3^Medical Service Section, The First Affiliated Hospital of Nanjing Medical University, Nanjing 210000, China; ^4^General Practice Department, The Geriatric Hospital of Nanjing Medical University, Nanjing 210000, China; ^5^Department of Rehabilitation Medicine, The First Affiliated Hospital of Nanjing Medical University, Nanjing 210000, China

## Abstract

**Background:**

This research is aimed at establishing and internally validating the risk nomogram of insulin resistance (IR) in a Chinese population of patients with polycystic ovary syndrome (PCOS).

**Methods:**

We developed a predictive model based on a training dataset of 145 PCOS patients, and data were collected between March 2018 and May 2019. The least absolute shrinkage and selection operator regression model was used to optimize function selection for the insulin resistance risk model. Multivariable logistic regression analysis was used to construct a prediction model integrating the function selected in the regression model of the least absolute shrinkage and selection operator. The predicting model's characteristics of prejudice, disease, and lifestyle were analyzed using the C-index, the calibration diagram, and the study of the decision curve. External validity was assessed using the validation of bootstrapping.

**Results:**

Predictors contained in the prediction nomogram included occupation, disease durations (years), BMI, current use of metformin, and activities. With a C-index of 0.739 (95 percent confidence interval: 0.644–0.830), the model showed good differentiation and proper calibration. In the interval validation, a high C-index value of 0.681 could still be achieved. Examination of the decision curve found that the IR nomogram was clinically useful when the intervention was determined at the 11 percent IR potential threshold.

**Conclusion:**

This novel IR nomogram incorporates occupation, disease durations (years), BMI, current use of metformin, and activities. This nomogram could be used to promote the estimation of individual IR risk in patients with PCOS.

## 1. Background

Among pregnant women, polycystic ovary syndrome (PCOS) is a more common disease that severely affects their physical and mental health [1]. Polycystic ovary syndrome is characterized by hyperandrogenemia and hyperinsulinemia [2]. Although insulin resistance and hyperinsulinemia are not the diagnostic criteria of PCOS, about 75% of PCOS women have the endocrine characteristics of insulin resistance [3].

The article "Predicting Risk of Insulin Resistance in a Chinese Population with Polycystic Ovary Syndrome: Designing and Testing a New Predictive Nomogram" was retracted in 2024. Reasons: signs of a paper mill; suspected computer-generated content; unreliable results or conclusions; concerns about the data.

In recent years, insulin resistance is considered as the main pathological feature of PCOS, including obese and thin PCOS women [4]. At the same time, insulin resistance (IR) is also the leading cause of the metabolic syndrome. At present, many studies have shown that nearly 50% of women with PCOS have metabolic syndrome (MS) [5]. Polycystic ovarian syndrome is therefore associated with an increased risk of type 2 diabetes and cardiovascular events [6]. However, insulin resistance is affected by multiple determinants such as patient-related factors (e.g., age, sex, employment, educational level, disease duration (years), body mass index (BMI), and waist-hip ratio (WHR)), disease-related factors (e.g., total cholesterol (TC), total glyceride (TG), low-density lipoprotein (LDL), hypertension, and current use of metformin), and lifestyle-related factors (e.g., sleeping time, mealtime, and activities).

Considering the risk of insulin resistance and many related risk factors, it is very important to find an accurate clinical prediction tool to predict the occurrence of insulin resistance. A sample of women with PCOS identified by the Rotterdam Consensus Workshop guidelines (2003) was assessed on whether insulin has resistance according to the homeostasis model assessment (HOMA) [1]. Based on HOMA, a predicted nomogram may have an impact on PCOS patients who may have IR. However, as far as we know, there is no research on this subject.

The goal of this research was to establish an accurate and easy predictive method for polycyclic ovarian syndrome, using features that were easily available to estimate the risk of occurrence.

## 2. Methods

### 2.1. Patients

Research approval was obtained from the Ethics Committee of the Obstetrics and Gynecology Hospital of Fudan University (approval no [2018]56). From March 2018 to May 2019, patients were recruited from Fudan University's Obstetrics and Gynecology Hospital, and they came from all over China. If they were 15-49 years old and met the PCOS guidelines of the Rotterdam Consensus Workshop (2003), the patients were included. All patients gave written informed consent, completed the lifestyle appraisal questionnaire, and took part in a 15-minute sports medical expert interview. The research does not include illiterate patients with severe cognitive impairment or severe physical disabilities. Patient characteristics of age, illness, and diagnosis were obtained from medical records. Insulin resistance was evaluated by HOMA-IR ([IR index = FPG (mmol/L) × FINS (mU/L)/22.5] ≥ 2.8) [7, 8].

The article "Predicting Risk of Insulin Resistance in a Chinese Population with Polycystic Ovary Syndrome: Designing and Testing a New Predictive Nomogram" was retracted in 2024. Reasons: signs of a paper mill; suspected computer-generated content; unreliable results or conclusions; concerns about the data.

### 2.2. Statistical Analysis

All results, including characteristics of populations, disease, and lifestyle, are expressed as a percentage of the count (percent). R software was used for statistical analysis (Version 3.6.1; https://www.R-project.org).

To select the best predictive features of risk factors from patients with PCOS, the least absolute shrinkage and selection operator (LASSO) [9, 10] approach for high-dimensional data compression is used [11, 12]. The characteristic of the nonzero coefficient in the cable regression model is selected [13]. Then, using multivariate logistic regression analysis, combined with the characteristics selected in the cable regression model, the prediction model is established. These characteristics are considered as odds ratios (or) with 95% confidence intervals (CI) and *P* values. The statistical significance level was bilateral. The model included the social demographic variables with a *P* value of 0.05, while the variables related to the characteristics of disease and lifestyle were included [7, 14, 15]. All the potential predictors were applied to build an IR risk prediction model by using the cohort. The correction curve was drawn to evaluate the correction of the insulin resistance nomogram. A significant test statistic shows that the model is not fully calibrated [16]. In order to quantify the discrimination of the insulin resistance nomogram, the C-index of Harrell was measured. The relative corrected C-index was calculated by bootstrapping verification (1000 bootstrap resampling) [17]. In order to determine the clinical usefulness of the insulin resistance nomogram, the decision curve approach was used to measure the net benefits of various threshold probabilities in the IRD cohort [18]. Net profit was determined by eliminating the proportion of all assumed positive individuals from the proportion of actual positive individuals and measuring the relative risk of abandoning interventions against the negative effects of ineffective interventions [19].

## 3. Results

### 3.1. Patients' Characteristics

A total of 145 patients attending our clinic completed the investigation from March 2018 to May 2019. Both patients were divided into groups of insulin resistance and noninsulin resistance (mean age 27.28 ± 4.45 years [range 15–39 years]) according to HOMA-IR. All patient data, including characteristics of demographics, disease, and lifestyle in both groups, are presented in Table 1.

### 3.2. Feature Selection

In demographic characteristics, disease, and lifestyle, 14 characteristics were reduced to five potential indicators based on 145 cohort patients (~3 : 1 ratio; Figures 1(a) and 1(b)) and were present in the LASSO regression model with nonzero coefficients. Such characteristics include occupation, disease period (years), BMI, existing metformin use, and behaviors (Table 2).

The article "Predicting Risk of Insulin Resistance in a Chinese Population with Polycystic Ovary Syndrome: Designing and Testing a New Predictive Nomogram" was retracted in 2024. Reasons: signs of a paper mill; suspected computer-generated content; unreliable results or conclusions; concerns about the data.

### 3.3. Development of an Individualized Prediction Model

The results of the study of logistic regression between occupation, period of disease (years), BMI, current metformin use, and behaviors are summarized in Table 2. A model was developed and presented as the nomogram including the above independent predictors (Figure 2).

### 3.4. Apparent Accuracy of the Cohort's IR Exposure Nomogram

In this cohort, the calibration curve of the IR risk nomogram for insulin resistance risk prediction for PCOS patients showed good agreement (Figure 3). For the sample, the C-index for the prediction nomogram was 0.739 (95 percent CI: 0.644–0.830) and was verified to be 0.681 by bootstrapping validation, indicating strong discrimination against the model. Apparent output in the IR risk nomogram presented an outstanding ability to predict.

### 3.5. Clinical Use

The IR nomogram's decision curve analysis is shown in Figure 4. The decision curve indicates that if the threshold likelihood of patients and doctors is greater than 11% and less than 70%, respectively, the use of the nonadherence nomogram to estimate drug nonadherence risk adds more benefits than the scheme. In this range, according to the IR risk nomogram, the net benefit can be compared with several overlaps.

## 4. Discussion

At present, nomograms have been widely used in the prognosis analysis of tumors and medicine [20]. Nomograms rely on a user-friendly digital interface, greater accuracy, and clearer interpretation of prognosis to help make better clinical decisions. Our research is the first to apply this nomogram to the treatment of PCOS and resistance to insulin.

We developed and validated a new predictive tool that uses five easily available variables to predict the risk of insulin resistance in patients with PCOS. Integrating risk factors of demography, disease, and lifestyle characteristics into an easy-to-use nomogram is helpful for the individual prediction of insulin resistance formation in patients with PCOS. If we can infer the patient who will have insulin resistance in the future through its related factors, we can screen out the high-risk population of insulin resistance, so as to gain a time window for clinical intervention and treatment. This study provides a predictive method for insulin resistance in patients with polycystic ovary syndrome that is relatively accurate. The queue's internal validation shows good differentiation and calibration capability; in particular, our high C-index in interval validation indicates that because of its fairly large sample size, the nomogram can be used extensively and accurately.

The article "Predicting Risk of Insulin Resistance in a Chinese Population with Polycystic Ovary Syndrome: Designing and Testing a New Predictive Nomogram" was retracted in 2024. Reasons: signs of a paper mill; suspected computer-generated content; unreliable results or conclusions; concerns about the data.

Similar to previous studies [21–23], in our study, about 69% of PCOS patients showed insulin resistance. In the analysis of risk factors, insulin resistance of PCOS patients is related to employment, the duration of disease, BMI, whether they take metformin at present, and the activity time. The nomogram shows that employment, duration of disease, BMI, whether metformin is taken at present, and activity time may be the key individual factors determining insulin resistance in PCOS patients [24, 25].

Among the five key factors related to insulin resistance of PCOS patients identified in this study, employment, BMI, and daily activity time are closely related to PCOS. Employment is closely related to insulin resistance. Several research investigated shift work with respect to hormone levels of reproduction [26]. These women are more likely to have shorter or longer lengths of menstrual cycles [27]. Our study also shows that women with PCOS in these workplaces have a greater proportion of insulin resistance. BMI, especially central obesity, is closely related to insulin resistance in many metabolic diseases. In our study, BMI is also the key factor of insulin resistance in PCOS patients. A sedentary lifestyle is the main cause of obesity, and lifestyle improvement, including diet and exercise, has been gradually recommended as the primary nondrug therapy for PCOS in recent years [28]. We investigated the daily life and rest time of PCOS patients, including sleep, diet, and activity time. We found that daily activity time is also a key factor for insulin resistance in patients. Metformin, as the first-line drug for PCOS treatment, has been proven to have the effect of increasing insulin sensitivity by many studies. Some studies have found that nearly 50% of women who sleep less than six hours have irregular menstrual cycles. In contrast, only 25% of women who sleep more than six hours have menstrual disorders [27, 29, 30]. They observed that there was a significant association of short sleep duration rather than shiftwork with changes in the length of the menstrual cycle. Other epidemiological studies have shown that repeated sleep deprivation at night can lead to insulin resistance and diabetes in healthy adults. However, in this study, sleep duration was not a significant factor in the insulin resistance of PCOS.

Insulin resistance is strongly associated with PCOS and MS. And insulin resistance in PCOS patients is closely related to the occurrence of cardiovascular complications. At present, although whether patients have insulin resistance can be measured, there is no tool to predict whether patients will have insulin resistance in the long term. Our goal is to establish a model to predict whether patients will have insulin resistance in the future. The development of insulin resistance risk prediction tools can improve the outcome of patients through individualized risk prediction and intervention. At the same time, we developed an effective risk prediction tool for insulin resistance to help clinicians pay more attention to significant factors, early treatment, and intervention from the perspective of factors to reduce the outcome of cardiovascular disease. It can also be used as a user guide in clinical research for the best choice of PCOS patients. For example, the nomogram created would direct researchers through clinical trials to select accurate patients with characteristics.

The article "Predicting Risk of Insulin Resistance in a Chinese Population with Polycystic Ovary Syndrome: Designing and Testing a New Predictive Nomogram" was retracted in 2024. Reasons: signs of a paper mill; suspected computer-generated content; unreliable results or conclusions; concerns about the data.

Therefore, for PCOS patients, the early prediction of insulin resistance has positive clinical significance for the treatment and prognosis of patients.

## 5. Limitations

Our current research also has some limitations. First of all, the data we collected may only represent some PCOS women. This cohort does not represent all Chinese PCOS patients. Second, not all possible factors that influence insulin resistance were included in the risk factor study. Some possible aspects of disobedience, such as social support and other facts, are not fully understood. Third, although the bootstrap test has thoroughly checked the robustness of our nomogram, the external testing cannot be conducted and its generality is unknown for other PCOS populations in other regions and countries. In a wider population, it needs to be evaluated externally.

## 6. Conclusion

This research established a relatively high accuracy new nomogram to help clinical staff understand the risk of insulin resistance in PCOS patients. Physicians and patients may take more necessary measures in controlling lifestyle and medical intervention through individual risk assessment. This nomogram requires external testing and further analysis to determine whether individualized therapy based on this nomogram will minimize related complications and improve the prognosis of polycystic ovary syndrome patients.

## Figures and Tables

**Figure 1:** Demographic and clinical feature selection using the LASSO binary logistic regression model. Notes: (a) the optimal parameter (lambda) in the lasso model is selected by the minimum criterion of five crossvalidations. The partial likelihood deviation (binomial deviation) curve and the logarithm (lambda) curve are drawn. Use 1se (1-SE standard) of minimum standard and minimum standard to draw a dashed vertical line at the best value. (b) LASSO coefficient profiles of the 22 features. According to the sequence of the logarithm (lambda), the coefficient profile is drawn. A fivefold crossvalidation is used to draw a vertical line at the selected value, where the optimal lambda produces five nonzero coefficients. Abbreviations: LASSO: least absolute shrinkage and selection operator; SE: standard error.

The article "Predicting Risk of Insulin Resistance in a Chinese Population with Polycystic Ovary Syndrome: Designing and Testing a New Predictive Nomogram" was retracted in 2024. Reasons: signs of a paper mill; suspected computer-generated content; unreliable results or conclusions; concerns about the data.

**Figure 2:** Developed IR nomogram. Note: the IR nomogram was developed in the cohort, with the employment, disease duration, BMI, current use of metformin, and activities.

**Figure 3:** Calibration curves of the IR nomogram prediction in the cohort. Notes: the *x*-axis represents the predicted IR risk. The *y*-axis represents the actual diagnosed IR. The diagonal dotted line represents a perfect prediction by an ideal model. The solid line represents the performance of the nomogram, of which a closer fit to the diagonal dotted line represents a better prediction.

**Figure 4:** Decision curve analysis for the IR nomogram. Notes: the *y*-axis measures the net benefit. The dotted line represents the IR risk nomogram. The thin solid line represents the assumption that all patients are IR. The thin, thick solid line represents the assumption that no patients are non-IR. The decision curve showed that if the threshold probability of a patient and a doctor is 11% and 70%, respectively, using this IR nomogram in the current study to predict insulin resistance risk adds more benefit than the intervention-all-patients scheme or the intervention-none scheme.

**Table 1:** Differences between demographic and clinical characteristics of IR and non-IR groups.

Demographic characteristics	*n*%		
	Insulin resistance (101)	Noninsulin resistance (44)	Total (145)
Age (years)			
<20	4 (66.67)	2 (33.33)	6 (4.14)
20-30	65 (66.33)	33 (33.67)	98 (67.59)
30-40	32 (78.05)	9 (21.95)	41 (28.29)
Education level			
Secondary (9-12 years)	39 (67.24)	19 (32.76)	58 (40.00)
Higher (>12 years)	62 (71.26)	25 (28.74)	87 (60.00)
Occupation			
Employed	45 (58.44)	32 (41.56)	77 (53.10)
Unemployed	56 (82.35)	12 (17.65)	68 (46.90)
Disease durations (years)			
0-1	25 (56.82)	19 (43.18)	44 (30.34)
1-5	63 (72.41)	24 (27.59)	87 (60.00)
5-10	12 (92.31)	1 (7.69)	13 (8.97)
>10	1 (100)	0 (0)	1 (0.69)
BMI			
≥28	69 (79.31)	18 (20.69)	87 (60.00)
≥24,<28	28 (59.57)	19 (40.43)	47 (32.41)
18.5-24	4 (40.00)	6 (60.00)	10 (6.90)
<18.5	0 (0)	1 (100)	1 (0.69)
WHR			
<0.8	16 (66.67)	8 (33.33)	24 (16.55)
≥0.8	85 (70.25)	36 (29.75)	121 (83.45)
Clinic characteristics			
TC			
Normal	93 (69.40)	41 (30.60)	134 (92.41)
Abnormal	8 (72.73)	3 (27.27)	11 (7.59)
TG			
Normal	59 (67.82)	28 (32.18)	87 (60.00)
Abnormal	41 (71.93)	16 (28.07)	58 (40.00)
LDL			
Normal	67 (67.67)	32 (32.32)	99 (68.28)
Abnormal	34 (73.91)	12 (26.09)	46 (31.72)
Hypertension			
Normal	77 (66.38)	39 (33.62)	116 (80.00)
Abnormal	24 (82.76)	5 (17.24)	29 (20.00)
Current use of metformin			
No	83 (72.81)	31 (17.19)	114 (78.62)
Yes	18 (58.06)	13 (41.94)	31 (21.38)
Lifestyle (day)			
Sleeping duration			
<6 h	28 (66.67)	14 (33.33)	42 (28.97)
≥6 h	73 (70.87)	30 (29.13)	103 (71.03)
Mealtime			
<30 min	42 (79.25)	11 (20.75)	53 (36.55)
≥30 min	59 (64.13)	33 (35.87)	92 (63.45)
Activities			
<30 min	62 (81.58)	14 (18.42)	76 (52.41)
≥30 min	39 (56.52)	30 (43.48)	69 (47.59)

The article "Predicting Risk of Insulin Resistance in a Chinese Population with Polycystic Ovary Syndrome: Designing and Testing a New Predictive Nomogram" was retracted in 2024. Reasons: signs of a paper mill; suspected computer-generated content; unreliable results or conclusions; concerns about the data.

**Table 2:** Prediction factors for IR in PCOS.

Intercept and variable	Prediction model		
	*β*	Odds ratio(95% CI)	*P* value
Intercept	1.099	3 (1.112-8.76)	0.035
Employment			
No	Reference		
Yes	0.606	1.832 (0.722-4.736)	0.203
Disease durations			
Disease durations (<1)	Reference		
Disease durations (1-5)	0.304	1.355 (0.574-3.154)	0.482
Disease durations (6-10)	1.363	3.91 (0.553-8.040)	0.239
Disease durations (>10)	13.862	—	0.992
BMI			
BMI (≥28)	Reference		
BMI (≥24, <28)	-0.551	0.576 (0.207-1.578)	0.284
BMI (18.5-24)	-1.178	0.308 (0.058-1.520)	0.152
BMI (<18.5)	-15.26	—	0.992
Current use of metformin			
No	Reference		
Yes	-0.937	0.392 (0.152-0.997)	0.049
Activities			
Activities < 30 min	Reference		
Activities ≥ 30 min	-0.468	0.627 (0.245-1.598)	0.325

## Data Availability

The datasets are available from the corresponding author on reasonable request.

## Abbreviations

PCOS: Polycystic ovary syndrome
IR: Insulin resistance
MS: Metabolic syndrome
BMI: Body mass index
WHR: Waist-hip ratio
TC: Total cholesterol
TG: Total glyceride
LDL: Low-density lipoprotein
LASSO: Least absolute shrinkage and selection operator
SE: Standard error.
